# Serum Cystatin C Level Monitoring for Intervention Opportunity of CBP in Children with Severe Sepsis

This article has been retracted.

**DOI:** 10.1155/2022/8571203

**Published:** 2022-06-29

**Authors:** Weikai Wang, Yi Qiang, Zhongbin Tao, Baowang Yang, Bin Yan, Xilong Chen, Ruifeng Xu

**Affiliations:** ^1^Department of PICU, Gansu Provincial Maternity and Child-Care Hospital, The First Clinical Medical College of Gansu University of Chinese Medicine, Lanzhou 730050, Gansu, China; ^2^Cardiovascular Diseases Center, Gansu Provincial Maternity and Child-Care Hospital, Lanzhou 730050, Gansu, China; ^3^Department of PICU, The First Hospital of Lanzhou University, Lanzhou 730000, Gansu, China; ^4^Department of PICU, The Second Hospital of Lanzhou University, Lanzhou 730030, Gansu, China; ^5^Department of PICU, Gansu Provincial Maternity and Child-Care Hospital, Lanzhou 730050, Gansu, China

## Abstract

**Objective:**

The aim of this study is to investigate the instruction value of the serum cystatin C (Cys C) level monitoring for intervention opportunity of continuous blood purification technology (CBP) in children with severe sepsis.

**Methods:**

67 children with severe sepsis in the pediatric intensive care unit (PICU) with CBP treatment were retrospectively selected from May 2016 to April 2020. According to the time intervals between the time point of serum Cys C level began to increase (>15 mg/L) and the time point of CBP began, all children were divided into group A (<24 h, 29 cases), group B (24–48 h, 22 cases), and group C (>48 h, 16 cases). The children's general characteristics, vital signs, biochemical parameters, acute physiology and chronic health evaluation (APACHE II), and sequential organ failure assessment (SOFA) scores were evaluated. The influence factors of prognosis of children with severe sepsis were analyzed by multivariate regression analysis.

**Results:**

The intervals between the time point of PICU hospitalization and the time point of CBP began and the times of CBP in group A were significantly more than those in group B and C (*P* < 0.05). There was no statistically significant duration of CBP among three groups (*P* > 0.05). After follow-up of 28 d, there was no significant difference on the occurrence of coagulation disorders and hypovolemic shock induced by CBP among three groups (*P* > 0.05). However, the mortality of children in group A was lower than that in group C (*P* < 0.05). Children in group A had lower APACHE II scores, SOFA scores, serum *K*+, blood urea nitrogen (BUN), serum creatine (SCr), partial pressure of carbon dioxide (PCO_2_), and higher partial pressure of oxygen (PO_2_) than those of children in group C after CBP. (*P* < 0.05). SOFA scores ≥5 after CBP treatment and the time intervals between the time point of serum Cys C level began to increase (>15 mg/L) and the time point of CBP began ≥24 h were the independent influence factors on the prognosis by multivariate regression analysis.

**Conclusion:**

There are significant evidences that continuous blood purification technology within 24 h of serum Cys C level may better control the condition of children with severe sepsis.

## 1. Introduction

Sepsis is one of the main critical illnesses in the pediatric intensive care unit (PICU), with a high in-hospital mortality rate, and more than 40% of children with sepsis will be accompanied by an acute kidney injury (AKI) [1]. Continuous blood purification (CBP) is a widely used technique for the extracorporeal circulation support therapy in PICU [2]. In 2012, the “Expert Consensus on Continuous Blood Purification for the Treatment of Severe Sepsis in Children” drafted by 18 Chinese experts proposed that CBP should be used for the treatment of severe sepsis in children. However, the timing of CBP intervention in children with severe sepsis has been controversial. Most scholars believe that early intervention of CBP can reduce the mortality of children with a septic acute kidney injury [3]. However, there is no consensus on the definition of “early”. Finding sensitive indicators to start CBP has always been a difficult problem for PICU doctors to solve. In adult patients with sepsis, serum creatinine (SCr) and 24-hour urine output are often used as indicators of CBP initiation [4]. However, the creatinine value of children varies at different ages and is susceptible to the interference of tubular secretion and other nonrenal factors [5]. As the urination of infants is often involuntary, the collection of urine from infant patients is difficult. Therefore, It is not accurate to use serum creatinine and 24h urine volume as indicators of CBP intervention, which may easily lead to missed diagnosis or delayed treatment. Serum cystatin C (Cys C) is a kind of endogenous small molecule protein, which is continuously expressed at a constant rate in various nucleated cells and excreted by the kidneys. It is considered to be a sensitive indicator of early renal injury [6]. Here, we studied the renal replacement therapy for children with severe sepsis under the guidance of serum Cys C levels and compared the efficacy of starting CBP at different times.

## 2. Materials and Methods

### 2.1. Clinical Data

The clinical data of 67 children with sepsis who received CBP treatment in the PICU of our hospital from May 2016 to April 2020 were retrospectively analyzed. Among them, 40 were male and 27 were female. The age ranged from 28 days to 12 years old, the average age was (5.27 ± 3.32) years old; blood/deep sputum specimens/pleural effusion were cultured in all the children, among which 41 cases were positive (12 cases of *Pseudomonas aeruginosa*, 7 cases of methicillin-resistant coagulase-negative staphylococci, 5 cases of methicillin-resistant *Staphylococcus aureus*, 5 cases of *Streptococcus pneumoniae*, 4 cases of *Klebsiella pneumoniae* subsp. ppneumonia, 3 cases of hemolytic streptococcus, 2 cases of *Escherichia coli*, 1 case of *Pseudomonas aeruginosa*, 1 case of *Enterococcus faecalis*, methicillin-resistant hemolytic grape 1 case of cocci), and the other 2 cases were positive for EB virus DNA.

#### 2.1.1. Diagnostic Criteria for Severe Sepsis

The diagnostic criteria were as follows: ①All children meet the diagnostic criteria for sepsis in the “China Guidelines for Diagnosis and Treatment of Severe Sepsis/Septic Shock (2014 Edition)” issued by the Chinese Society of Critical Care Medicine: the presence of definite or suspected systemic inflammatory response syndrome systemic inflammatory response syndrome (SIRS) and typical symptoms of infection: body temperature >38°C or <36°C, tachycardia, dyspnea, lethargy, edema, hyperglycemia (without history of diabetes), abnormal blood routine index, hypotension, organ dysfunction, hyperlactatemia, etc. In addition, combined with cerebral edema, liver failure, acute respiratory distress syndrome (ARDS), severe acid-base imbalance and electrolyte imbalance, conventional therapy is difficult to correct. ②with persistent involvement of more than one organ failure for more than 48 hours or local complications; and ③sequential organ failure assessment (SOFA) ≥3 points; acute physiology and chronic health evaluation II (APACHE II) score ≥8 points; modified CT severity index score ≥4 point. All patients sign an informed consent form.

#### 2.1.2. Inclusion Criteria

The inclusion criteria were as follows: ①Children who meet the diagnostic criteria for severe sepsis in “China Guidelines for Diagnosis and Treatment of Severe Sepsis/Septic Shock (2014 Edition)”. ②Age ≤18 years old. ③Admission to hospital within 48 hours after onset. ④Patients who continue to receive CBP treatment for more than 24 hours.

#### 2.1.3. Exclusion Criteria

The exclusion criteria were as follows: ①Children who do not meet the above inclusion criteria. ②Children with a history of renal transplantation or renal replacement therapy. ③Persons with glomerulonephritis, interstitial nephritis, renal vasculitis, and end-stage renal disease. ④Combined kidney tumors, immune system, blood system diseases, and severe bleeding tendency.

### 2.2. Treatment

#### 2.2.1. Conventional Treatment

All children were treated in accordance with the “Chinese Guidelines for Diagnosis and Treatment of Severe Sepsis/Septic Shock (2014 Edition)”, including antibiotics within 1 hour of diagnosis, completion of fluid resuscitation within 6 hours, maintenance of acid-base balance and electrolyte balance, early body fluid resuscitation, strengthen parenteral nutrition, etc.

#### 2.2.2. CBP Treatment

If the child's condition is relieved after conventional treatment or the following indications occur, CBP treatment should be given immediately: ① Severe hyperkalemia: serum potassium >6.5 mmol/L. ② Water intoxication: Heart failure, severe hyperkalemia caused by excessive volume overload hypertension or pulmonary edema. ③ Severe metabolic acidosis: blood pH < 7.20, blood HCO_3_- <12 mmol/L. ④ Serum urea nitrogen (BUN) >28.7 mmol/L (80 mg/dl) or SCr >442 *μ*mol/L (6 mg/dl). ⑤ Decreased urine output: anuria for 2 days or oliguria for more than 4 days. Femoral vein or internal jugular vein catheterization was performed using the Seldinger technique, vascular access was established, and the Prismaflex (Gambro, Sweden) or BM25 (Baxter, USA) continuous blood purification system was used, 16–18 *G* single lumen (≤1 year old), 6.5–11.5 *F* single-needle double-lumen tube (>1 year old), and child-type tube. Children with a body weight <20 kg should choose 0.2–0.4 m^2^ polysulfone membrane, those weighing 20–30 kg should choose 0.4–0.8 m^2^ polysulfone membrane, and those above 30 kg should choose 0.8–1.0 m^2^ polysulfone membrane. The hemofiltration machine produces the replacement fluid online. The blood flow rate is 3–5 ml/(kg h), the dialysate is 30–50 ml/(kg h), the pre-replacement: the post-replacement ≈1 : 2, and the dehydration amount is 0–2 ml/(kg h); the amount of ultrafiltration is adjusted according to the condition and clinical needs of the child. Each child is treated 1-2 times according to the condition. In addition, low-molecular-weight heparin anticoagulation or low-molecular-weight heparin anticoagulation can be selected according to the condition of the child, and no heparin treatment can be used when there is a tendency to bleeding.

### 2.3. Monitoring and Grouping of the Serum Cys C Level

Daily blood samples were collected from children, and serum Cys C levels were remeasured by particle-enhanced transmission immunoturbidimetry. The time interval between the start of serum Cys C level and the initiation of CBP was recorded, and 67 patients were divided into group A (<24 h, 29 cases), group B (24–48 h, 22 cases), and group C (>48 h, 16 cases).

### 2.4. Indicator Observation

#### 2.4.1. General Clinical Data

The gender and age of the children were included, and the duration of CBP (d) and the 28-day mortality were recorded.

#### 2.4.2. Vital Signs

The body temperature, heart rate, respiratory rate, and urine output of the children before and 48 hours after CBP treatment were recorded.

#### 2.4.3. Biochemical Parameters

Blood routine, liver function electrolytes, arterial blood gas analysis, and other indicators were included.

#### 2.4.4. Disease Severity Score

The APACHE II score and SOFA score of the children were evaluated depending on the daily condition of the children.

### 2.5. Statistical Processing

Input the data into SPSS17.0 statistical software for processing and analysis, the measurement data conforming to the normal distribution are expressed as (*χ* ± *s*), the data between the two groups are compared by an independent sample *t*-test, and the same group at different time points. The variables were compared using paired samples *t*-test; data comparison between multiple groups was performed using one-way ANOVA analysis. The enumeration data were expressed as (%), and the *χ*^2^ test was used, and *P* < 0.05 was considered to be statistically significant.

## 3. Results

### 3.1. Comparison of Baseline Data of the Three Groups of Children

The basic information, vital signs, and main biochemical parameters of the children in group A, group B, and group C at admission were compared. The age, gender composition, heart rate, APACHE II score, SOFA score, basal body temperature, urine volume, alanine transaminase (ALT), aspartate aminotransferase (AST), serum HCO_3−_, serum potassium level, BUN, SCr, partial pressure of oxygen (PO_2_), partial pressure of carbon dioxide (partial pressure) of carbon dioxide (PCO_2_), oxygenation index (PO_2_/FiO_2_), and etiological test results were basically the same, with no statistical difference (*P* > 0.05), which was comparable as shown in Table 1.

### 3.2. CBP Treatment of Children in the Three Groups

The time interval of CBP intervention in the three groups was 2 h–96 h after admission, and the total treatment time was 10 h–76 h. The time from admission to CBP intervention, the number of interventions, and the treatment time were compared among the three groups. As for the time of CBP intervention and the number of interventions, it was found that the children in groups B and C were significantly more than those in group A, and the difference was statistically significant (*P* < 0.05) as shown in Table 2.

### 3.3. Comparison of Clinical Outcomes of the Three Groups of Children

During the 28-day follow-up, there was no significant difference in the incidence of complications such as coagulation dysfunction and hypovolemic shock among the three groups (*P* > 0.05). The mortality rate of children in group C and group B was slightly higher than that of children in group A and there was a statistical difference *P* < 0.05. For children with coagulation dysfunction, plasma, platelets, and protamine were transfused according to the situation, and the coagulation function gradually returned to normal. For 1 child with embolism, thrombolysis with urokinase was administered in time, and heparin sodium and dextran were used for anticoagulation without serious consequences. For the 3 children with hypovolemic shock, normal saline volume expansion was given first, which was quickly corrected and then continued CBP therapy as shown in Table 3.

### 3.4. Changes of Vital Signs and Biochemical Indexes in the Three Groups of Children after Treatment

After CBP intervention, compared the vital signs and main biochemical parameters of the children in groups A, B, and C at admission, the heart rate, basal body temperature, serum HCO_3−_, ALT, AST, and PO_2_/FiO_2_ of the three groups were basically the same, there was no statistical difference (*P* > 0.05); but after CBP intervention, the APACHE II score, SOFA score, serum potassium level, BUN level, SCr level, and PCO_2_ value of the children in group A were significantly lower than those in the children in group C, and the difference was statistically significant (*P* > 0.05). Meanwhile, after CBP intervention, the APACHE II score, SOFA score, serum potassium level, BUN level, SCr level, and PCO_2_ value of the children in group A were also significantly lower than those in the children in group B. However, the PO_2_ value was higher than that of the children in group C, indicating the recovery rate of renal function in children with sepsis, and the difference was statistically significant (*P* < 0.05) as shown in Table 4.

### 3.5. Analysis of Factors Affecting the Prognosis of Children

Taking the treatment outcome of the children as the dependent variable (death was assigned a value of 1 and survival was assigned a value of 0), and the above variables with statistical differences after CBP intervention were used as independent variables; the forward stepwise (conditional) regression model was used for multivariate analysis. The results showed that the SOFA score ≥5 points after CBP intervention and the time from serum Cys C elevation to CBP intervention ≥24 hours were independent risk factors affecting the prognosis of children (*P* < 0.05). The prediction accuracy of the regression equation was 72.35%. Hosmer and Lemeshow Test was used to test the fit of the equation. There was no deviation between the fitted equation and the real equation (*P*=0.764). As shown in Table 5.

## 4. Discussion

Sepsis is one of the common critical illnesses in PICU with a complex etiology and rapid disease progression. In-hospital mortality is particularly high in children with severe sepsis. In recent years, with the maturation and standardization of CBP treatment technology, its application has become more and more extensive. It has not only been limited to the treatment of children with acute kidney injury but has gradually expanded to the application of various critical cases in the PICU, including the treatment of patients with severe sepsis. Increasing attention has been paid to the treatment of children [7]. In the past, most scholars believed that the initial indication of CBP treatment was acute kidney damage, such as serum potassium concentration higher than 6.5 mmol/L, pulmonary edema, heart failure, and sudden increase in blood pressure, or only when symptoms of uremia appeared. CBP [8]. However, because many clinical indicators in children vary with age and weight, there is some uncertainty. Especially in infants, vital signs and blood biochemical indicators vary greatly from those of adults, and it is difficult to collect urine, making the timing of initiation of CBP still highly controversial. l.

Serum Cys C belongs to a class of small molecule endogenous cystinase inhibitors. Unlike SCr, Cys C is almost exclusively secreted constantly by nucleated cells and excreted by the kidneys, with stable expression in peripheral blood and less interference from nonrenal factors [9]. Blood samples are easy to obtain, and the detection operation is simple and fast, and it is currently widely used in clinical practice. However, most studies focused on the changes of serum Cys C levels before and after CBP treatment, and few studies have evaluated the value of serum Cys C as the basis for CBP initiation in children with sepsis. Scholars such as Al-Beladi [10] have found through experiments that serum Cys C can diagnose acute renal injury 1.5 d–2 d earlier than SCr. Moradkhani et al. [11] also confirmed that Cys C can be used as an early diagnostic indicator of acute kidney injury associated with sepsis in children. In this study, we divided 67 children with severe sepsis into three groups according to the time interval from the time point of serum Cys C >15 mg/L to the time point of CBP initiation. The data, vital signs, main biochemical indicators (including SCr, BUN), and etiological test results were basically consistent and comparable. All the children received CBP intervention, the earliest was 2 hours after admission and the latest was 96 hours after admission. The total treatment time was 10 hours and 76 hours. The frequency was significantly more than that of group A children. In addition, after CBP intervention, the APACHE II score, SOFA score, serum potassium level, BUN level, SCr level, and PCO_2_ value in group A were significantly lower than those in group C, while the PO_2_ value was higher than that in group C. This indicated that when the serum creatinine, blood urea nitrogen, and other indicators were at the same level in the three groups, the shorter the time interval between the time point of serum Cys C elevation and the initiation of CBP, the higher the recovery rate of renal function in children with sepsis. This is basically consistent with the research conclusions of Hou et al. [12] Hou indicates that monitoring serum Cys C levels has an important guiding value for the clinical treatment of patients with sepsis complicated with multiple organ dysfunction and suggest that patients with elevated serum Cys C levels have an important guiding value suggesting that a good prognosis can be obtained with continuous renal replacement therapy within 48 hours.

In order to remove inflammatory mediators, cytokines, or endotoxins as soon as possible and prevent further deterioration of organ function, many foreign scholars recommend starting CBP therapy within 24 hours after admission to the ICU [13]. However, some multicenter clinical studies have confirmed that early continuous blood purification cannot significantly improve blood inflammatory indicators and prognosis in children with severe sepsis, but it has certain effects on improving oxygenation and tissue metabolism, and shortening the length of stay in PICU. Influence [14]. Therefore, the so-called early concept cannot simply be defined as the time interval between admission to the PICU and initiation of CBP. In this study, we took the time interval from the time point of serum Cys C level>15 mg/L to the time point of CBP initiation <24 h as the early treatment group (i.e., group A) and found that the mortality rate of children in group A was significantly lower at 28 days in group C, and the difference was statistically significant. It is suggested that taking the time of serum Cys C elevation as a reference index for starting CBP therapy has a high clinical outcome value. Subsequently, we further analyzed the multivariate logistic regression and found that the time interval between the time point of CBP intervention and the time point of SOFA score ≥5 and serum Cys C level >15 mg/L to the time point of CBP initiation was ≥24 hours was an independent risk factor affecting the prognosis of children. The APACHE II scoring system and the SOFA scoring system are the most commonly used quantitative assessment tools for nonspecific disease severity in clinical practice and are recognized and confirmed by most critical care medicine experts at home and abroad. However, the APACHE II scoring system is complex, and the assessment content includes the disease at the time of onset and the previous health status, and the clinical operability is poor, especially for critically ill children, it cannot make rapid, timely, and accurate judgments. In comparison, the SOFA scoring system is simple to operate, easy to collect data, and can quickly and effectively evaluate the renal function of children. Therefore, we suggest that the SOFA score and the time interval from the time point of serum Cys C level >15 mg/L to the time point of CBP initiation should be prioritized for children with severe sepsis as predictors of clinical outcome at 28 days.

In conclusion, this study found that continuous blood purification therapy can help improve the vital signs and renal function damage in children with severe sepsis, and CBP interventional therapy within 24 hours after the serum Cys C starts to rise is more effective. It shows that the serum Cys C level is expected to clinically guide the timing of starting CBP therapy in children with severe sepsis.

## Figures and Tables

**Table 1:** Comparison of basic clinical data, vital signs, and main biochemical parameters of the three groups of children on admission.

Index	Group A (*n* = 29)	Group B (*n* = 22)	Group C (*n* = 16)	*F*/*χ*^2^	*P* value
Old (year)	5.12 ± 3.14	5.31 ± 2.72	5.23 ± 3.59	0.024	0.977
Male/female	17/12	14/8	9/7	0.235	0.889
Heart rate (bpm)	107.41 ± 14.29	112.65 ± 17.20	104.72 ± 16.31	1.290	0.282
APACHE II score	25.93 ± 5.54	23.86 ± 5.75	23.90 ± 6.23	1.039	0.360
SOFA score	9.24 ± 2.37	9.08 ± 2.45	8.81 ± 2.92	0.148	0.862
Basal body temperature (°C)	37.91 ± 0.80	37.82 ± 0.81	37.89 ± 0.76	0.084	0.920
24 h urine output (mL)	1357 ± 1026	1185 ± 835	1039 ± 968	0.602	0.551
HCO_3_^−^ (mmol/L)	16.38 ± 4.85	16.11 ± 4.34	15.49 ± 5.26	0.179	0.837
ALT (U/L)	559.28 ± 411.46	517.97 ± 390.16	530.82 ± 375.23	0.074	0.929
AST (U/L)	662.21 ± 617.48	656.15 ± 633.80	629.24 ± 598.37	0.020	0.980
BUN (mmol/L)	20.91 ± 9.10	16.65 ± 9.48	17.82 ± 10.70	1.330	0.272
SCr (*μ*mol/L)	282.73 ± 79.42	245.23 ± 99.47	240.79 ± 113.42	1.437	0.245
Serum potassium (mmol/L)	4.78 ± 0.97	4.11 ± 0.85	4.42 ± 1.05	3.129	0.051
PO_2_ (mmHg)	87.45 ± 37.84	95.86 ± 35.89	107.95 ± 39.49	1.539	0.222
PCO_2_ (mmHg)	36.72 ± 13.29	32.57 ± 9.87	35.11 ± 11.23	0.778	0.464
PO_2_/FiO_2_ (mmHg)	205.78 ± 121.96	217.86 ± 98.59	244.53 ± 118.40	0.598	0.553

APACHE II: acute physiology and chronic health evaluation; SOFA: sequential organ failure assessment; ALT: alanine aminotransferase; AST: aspartate aminotransferase; BUN: blood urea nitrogen; SCr: serum creatinine; PO_2_: partial pressure of blood oxygen; PCO_2_: partial pressure of carbon dioxide; PO_2_/FiO_2_: oxygenation index.

**Table 2:** Treatment of CBP in the three groups of children.

Group	Intervention time of CBP (‾*χ* ± *s*, h)	2 CBP interventions (cases, %)	Length of CBP treatment (‾*χ* ± *s*, h)
Group A (*n* = 29)	11.30 ± 5.81	0	45.10 ± 19.83
Group B (*n* = 22)	32.77 ± 6.57^a^	5 (22.73)^a^	47.24 ± 23.25
Group C (*n* = 16)	52.46 ± 5.34^ab^	5 (31.25)^a^	44.64 ± 23.87
*F*	254.931	9.500	0.083
*P* value	0.000	0.009	0.920

Compared with group A, ^a^*P* < 0.05; compared with group B, ^b^*P* < 0.05.

**Table 3:** Comparison of clinical outcomes and complications among the three groups of children (cases, %).

Group	Death	Coagulation disorders	Embolism	Hypovolemic shock
Group A (*n* = 29)	6 (20.69)	3 (10.34)	0	0
Group B (*n* = 22)	10 (45.45)	5 (22.73)	0	1 (4.55)
Group C (*n* = 16)	9 (56.25) a	5 (31.25)	0	1 (6.25)
*F*	7.887	3.113	*—*	1.666
*P* value	0.019	0.211	—	0.435

Compared with group A, ^a^*P* < 0.05.

**Table 4:** Comparison of vital signs and main biochemical parameters of the three groups of children after treatment.

Index	Group A (*n* = 29)	Group B (*n* = 22)	Group C (*n* = 16)	*F*	*P* value
Heart rate (bpm)	82.81 ± 11.79	87.37 ± 14.98^a^	98.39 ± 14.72^ab^	6.794	0.002
Apache II score	9.86 ± 4.10	13.32 ± 4.53^a^	14.75 ± 4.45^a^	7.751	0.001
SOFAscore	4.39 ± 1.94	5.73 ± 2.10^a^	6.52 ± 2.29^a^	5.991	0.004
Basal body temperature (°C)	37.31 ± 0.56	37.39 ± 0.61	37.40 ± 0.65	0.164	0.849
HCO_3_- (mmol/L)	24.22 ± 5.95	24.07 ± 6.86	22.49 ± 7.10	0.398	0.673
ALT (U/L)	177.38 ± 179.84	186.24 ± 157.58	210.43 ± 148.06	0.208	0.813
AST (U/L)	295.86 ± 211.50	324.19 ± 185.47	330.79 ± 195.25	0.205	0.815
BUN (mmol/L)	10.18 ± 4.17	12.63 ± 5.06	14.81 ± 4.73^a^	5.425	0.007
SCr (*μ*mol/L)	86.89 ± 50.33	125.61 ± 43.78^a^	162.78 ± 61.25^ab^	11.739	0.000
Serum potassium (mmol/L)	1.27 ± 0.76	1.65 ± 0.72*∗*	1.99 ± 0.90^a^	4.548	0.014
PO_2_ (mmHg)	214.32 ± 38.59	200.57 ± 32.47	179.34 ± 51.30^a^	3.916	0.025
PCO_2_ (mmHg)	10.45 ± 7.58	15.28 ± 9.02^a^	20.76 ± 8.17^a^	8.270	0.001
PO_2_/FiO_2_ (mmHg)	347.15 ± 138.49	310.54 ± 107.92	256.57 ± 140.34	2.522	0.088

APACHE II: acute physiology and chronic health evaluation; SOFA: sequential organ failure assessment; ALT: alanine aminotransferase; AST: aspartate aminotransferase; BUN: blood urea nitrogen; SCr: serum creatinine; PO_2_: partial pressure of blood oxygen; PCO_2_: partial pressure of carbon dioxide; PO_2_/FiO_2_: oxygenation index; compared with group A, ^a^*P* < 0.05; compared with group B, ^b^*P* < 0.05.

**Table 5:** Multivariate logistic regression analysis affecting the outcome of children.

Influencing factors	*B*	SE	Walds	d*f*	Sig.	Exp (B)
SOFA score ≥5	0.237	0.051	6.889	1	0.007	1.258
From serum Cys C increasing to intervention of CBP ≥24 h	0.774	0.123	23.165	1	0.000	1.457
Constant	0.376	1.218	0.092	1	0.764	1.443

APACHE II: acute physiology and chronic health evaluation; SOFA: sequential organ failure assessment; Cys C: cystatin C; CBP: continuous blood purification.

## Data Availability

The data used and/or analyzed during the current study are available from the corresponding author upon request.
